The article "Comparison of Curative Effect between PFNA and PCCP in the Treatment of Femoral Intertrochanteric Fractures" was retracted in 2024. Reasons: signs of a paper mill; suspected computer-generated content; unreliable results or conclusions; concerns about the data.

# Comparison of Curative Effect between PFNA and PCCP in the Treatment of Femoral Intertrochanteric Fractures

**DOI:** 10.1155/2022/5957025

**Published:** 2022-08-13

**Authors:** Buxin Fan, Hansen Xiao, Peng Wu, Yao Du

**Affiliations:** Department of Orthopaedics, Daxing Teaching Hospital, Capital Medical University, Beijing 102600, China

## Abstract

**Objective:**

To compare and analyze the clinical efficacy of proximal femoral nail anti-rotation (PFNA) and percutaneous compression plate (PCCP) for minimally invasive treatment of femoral intertrochanteric fractures.

**Methods:**

A retrospective analysis of 98 patients with femoral intertrochanteric fractures admitted to our hospital from January 2019 to December 2020 was used as the research object, and they were divided into PFNA group and PCCP group according to different treatment methods, with 51 cases and 47 cases. The intraoperative and postoperative indicators were compared between the two groups of patients.

**Results:**

There was no significant difference in the operative time, postoperative fracture healing time, and Harris score of hip joint function between the two groups (*t* = −1.43, 1.86, 1.63; *P* > 0.05). Compared with the PFNA group, the intraoperative blood loss and postoperative drainage volume in the PCCP group were lower than those in the PFNA group (*t* = 11.38, 9.66; *P* < 0.05). Compared with the PFNA group, the time of weight-bearing in the PCCP group was longer than that in the PFNA group (*t* = −2.23, *P* < 0.05). The total incidence of postoperative complications was 7.84% in the PFNA group and 10.64% in the PCCP group, and there was no significant difference between the two groups (*P* > 0.05).

**Conclusion:**

The PFNA and PCCP are both effective measures for the clinical treatment of intertrochanteric fractures, and internal fixation should be reasonably selected according to the specific conditions of the patients.

## 1. Introduction

In clinical practice, femoral intertrochanteric fracture is one of the most common diseases in orthopedics, which refers to the fracture between the large and small intertrochanteric of the femur. It is mostly caused by indirect external force and usually manifests as comminuted fracture, and its clinical incidence is increasing year by year [1]. The condition is more common in the elderly. Because the elderly patients' own body bones are relatively loose and most elderly patients often have other diseases, if their intertrochanteric fractures are not treated in time, staying in bed for a long time may increase the risk of complications [2, 3]. The clinical treatment of femoral intertrochanteric fractures is the first choice for surgical treatment. The intraoperative fixation methods include intramedullary fixation and extramedullary fixation. The former is represented by proximal femoral nail anti-rotation (PFNA), and the latter is represented by percutaneous compression plate (PCCP) [4]. The two are the hot spots in the treatment of femoral intertrochanteric fractures. This study compared and analyzed the clinical therapeutic effects of PFNA and PCCP for minimally invasive treatment of femoral intertrochanteric fractures and provided a theoretical basis for clinical surgical treatment. The report is as follows.

## 2. Objects and Methods

### 2.1. Research Objects

A retrospective analysis of 98 patients with femoral intertrochanteric fractures admitted to our hospital from January 2019 to December 2020 was used as the research object. Inclusion criteria were as follows: no other systemic diseases; all patients were able to walk independently or with crutches before fracture. Pathological fracture cases and cases with surgical contraindications were excluded. According to different treatment methods, the patients were divided into PFNA group and PCCP group, with 51 cases and 47 cases, respectively. All patients were diagnosed with intertrochanteric fractures by X-ray examination. Among 98 patients, there were 51 males and 47 females, aged 29–83 years, with an average age of 68.13 years. The causes of injury include 17 cases of car accidents, 16 cases of high-altitude falling, and 65 cases of crash. The specific types of fractures were divided into 31 patients with type A1, 34 patients with type A2, and 33 patients with type A3. There was no significant difference in the general data of the two groups of patients (*P* > 0.05), and they were comparable. The general data of the two groups of patients are shown in Table 1. This study was approved by the ethics committee of the hospital, and all participants gave informed consent and signed the informed consent form.

### 2.2. Surgical Methods

All operations were performed by the same operator. ①Surgical methods of PFNA group: the patients underwent combined spinal-epidural anesthesia, the patient was placed in a supine position, and the affected hip was adducted and flexed for 30°. The C-arm X-ray machine closed the reduction. After the reduction was satisfactory, the towel was routinely disinfected, and a longitudinal incision was made at 3 cm above the greater trochanter to expose the top of the greater trochanter. The slotting device was used to slot in a 6-degree abduction position. Insert the guide needle into the femoral medullary cavity, enlarge the medulla, screw in the PFNA main nail, and make a longitudinal incision 2 cm downward from the bottom of the patient's greater trochanter. A guide needle was inserted through the center of the femoral neck, and after the position of the guide needle was confirmed, a spiral blade with appropriate length was inserted along the guide needle, and the distal screw was locked under the guidance. After the fracture position of the patient was checked and fixed, the tail cap was installed, and the incision of the patient was washed with physiological saline to complete the suture. ②Surgical method of PCCP group: the patients underwent combined spinal-epidural anesthesia, the patient was placed in a supine position, and the operation was performed under a C-arm X-ray machine. An incision of about 3 cm in length was made at the major trochanter, and a second incision about 2 cm was made after the steel plate was inserted. A percutaneous bone hook was inserted into it and fixed to a steel plate guide needle, and the length of the screw in the neck was measured. After the measurement, the first screw was placed in the femoral neck of the patient up to the lower part of the cartilage tissue of the femoral head. After the main sleeve was removed, the second incision was drilled to fix three backbone screws. Two femoral neck screws and other femoral shaft screws were completed by the same method. Under the fluoroscopy of C-arm X-ray equipment, the incision was washed and drainage tube was placed to complete the incision suture. ③After operation, routine ECG monitoring was performed in the two groups until the vital signs were basically normal, antibiotics were applied, and low molecular weight heparin sodium was given to the patients. Medical staff guided patients to exercise for rehabilitation.

### 2.3. Observation Items

Intraoperative indicators (operation time and intraoperative blood loss) and postoperative indicators (postoperative drainage volume, postoperative fracture healing time, time of weight-bearing, and postoperative Harris score of hip joint function) were compared between the two groups. Patients in the two groups were followed up for 12 months by telephone, Internet platform, and outpatient review. The complications were observed and counted.

### 2.4. Harris Hip Function Score [5]

At 12 months after operation, Harris hip function was evaluated from four aspects: pain (44 points), function (47 points), deformity (4 points), and range of motion (5 points). The scores of each item were cumulatively superimposed. The total score is 100 points, 90–100 points were considered excellent, 80–89 points were considered good, 70–79 points were considered average, and <69 points were considered poor.

### 2.5. Statistical Methods

SPSS 19.0 statistical software was used for analysis. Measurement data were represented by “ $\bar{x}\pm s$,” and *t*-test was used for comparison between groups; enumeration data were represented by “%,” and *χ*^*2*^ test was used for comparison between groups, and *P* < 0.05 was considered statistically significant.

## 3. Results

### 3.1. Comparison of Intraoperative Indicators between the Two Groups

There was no significant difference in the operative time between the two groups (*t* = −1.43, *P* > 0.05). The intraoperative blood loss and postoperative drainage volume in the PFNA group were significantly higher than those in the PCCP group (*t* = 11.38, *t* = 9.66, *P* < 0.05), as shown in Table 2. A typical case is shown in Figure 1.

### 3.2. Comparison of Postoperative Indicators between the Two Groups

There was no significant difference in fracture healing time between the two groups (*t* = 1.86, *P* > 0.05). The time of weight-bearing in the PCCP group was longer than that in the PFNA group, and the difference was statistically significant (*t* = −2.23, *P* < 0.05). There was no significant difference in hip function scores between the two groups (*t* = 1.63, *P* > 0.05), as shown in Table 3.

### 3.3. Comparison of Postoperative Complications between the Two Groups

The total incidence of postoperative complications was 7.84% in the PFNA group and 10.64% in the PCCP group, and there was no significant difference between the two groups (*P* > 0.05), as shown in Table 4.

## 4. Discussion

In clinical practice, the fracture from the base of the femoral neck to the area above the lesser trochanter is called intertrochanteric fracture. It is the most common type of fracture in the current clinical practice, and it is more common in the elderly. However, because the elderly patients are often accompanied by osteoporosis symptoms, their body resistance is gradually declining, and most of them are often complicated with basic systemic diseases, if they are not treated in time, prolonged bed rest can be complicated by diseases such as decreased cardiopulmonary function, which seriously threatens the life safety of elderly patients [6–8]. The clinical treatment of patients with intertrochanteric fractures generally follows the principles of minimal perioperative trauma, easy postoperative recovery, high safety, and mechanical stability [9]. At present, early surgical reduction and internal fixation are preferred. The common internal fixation methods include intramedullary fixation system and extramedullary nail plate system. The former is represented by PFNA, which has the advantages of less surgical trauma, less postoperative complications, and favorable prognosis [10]. The latter is represented by PCCP, which has the advantages of convenient operation and firmness, but its surgical trauma is relatively large, the postoperative healing time is relatively long, and the postoperative complications are relatively high [11].

The PFNA surgical treatment method can complete the corresponding material design according to the specific force principle of the patient's hip joint, which is closer to the patient's negative gravity line, which promotes the patient's load force transmission, and the overall diameter of the main nail is relatively small. Therefore, the joint stability and anti-rotation resistance of the treatment are increased to a certain extent [12, 13]. In PFNA, its force transmission is internal expansion and extrusion, so that the medial and lateral sides of the femur can bear the stress in a balanced manner. It has good biomechanical properties and can effectively prevent femoral shaft fractures. Its distal end is tilt-locked, which can reduce the risk of distant fractures [14]. In addition, the helical blade is operated after the guide needle is inserted into the femoral head, which can effectively increase the contact surface between the patient's head and neck screw and the cancellous bone and compress the cancellous bone, thereby preventing the loss of bone mass, and has a good effect on elderly patients with osteoporosis [15]. PCCP is a new type of internal fixation nail plate system in the current clinical practice. It is a minimally invasive surgery based on dynamic hip screws. The amount of postoperative blood loss, with a good fixation position, can effectively prevent the occurrence of lateral cortical fractures in patients and can effectively relieve postoperative pain [16]. Because the treatment method is biaxial fixation and has a certain sliding compression effect, it can increase the overall stability of the fracture end. However, in the treatment of PCCP, because the femoral neck of the patient is relatively narrow, the number of fixed distances between screws is limited. In addition, this treatment method is an extramedullary fixation method and is not suitable for patients with severe comminuted fractures and reverse trochanteric fractures. Therefore, this internal fixation method has some limitations [17]. In comparison, PFNA's internal fixation has higher requirements on the reduction of trochanteric fractures than PCCP internal fixation. PFNA requires good reduction before surgery; otherwise, the fracture site will be easily separated when the spiral blade is inserted. Previous studies have reported that PFNA surgery is more suitable for unstable intertrochanteric fractures with osteoporosis, while PCCP surgery is more suitable for some patients with basic diseases and poor physical condition [18].

This study showed that the intraoperative blood loss and postoperative drainage volume in the PCCP group were significantly smaller than those in the PFNA group mainly because the PCCP group was a minimally invasive operation, and the trauma was significantly smaller than that in the PFNA group. Therefore, PCCP is suitable for patients with poor physical condition and relatively low surgical tolerance. Some researchers [19] found that the intraoperative blood loss in the PCCP group was significantly lower than that in the PFNA group, which was consistent with the results of this study. In addition, this study found that the weight-bearing time of the PFNA group was shorter than that of the PCCP group. Due to the short force arm of the PFNA fixation and good biomechanical properties and the fact that its distal end is tilt-locked, it can reduce the risk of distant fractures.

This study showed that the total incidence of postoperative complications in PFNA group was 7.84%, and that in PCCP group was 10.64%. The incidence of postoperative complications in PFNA group was lower than that in PCCP group, but there was no significant difference between the two groups. This is consistent with the results reported by Arirachakaran et al. [20]. This is mainly due to the fact that PFNA internal fixation has less damage to surrounding soft tissue, less bleeding, less interference with fracture blood supply, and less loss of osteogenic factors in the fracture end hematoma, so the incidence of postoperative complications is low. However, PCCP is related to the longer operation time, more intraoperative blood loss, and extensive dissection of the fracture end, which increases the risk of infection.

In conclusion, the PFNA and PCCP are both effective measures for the clinical treatment of intertrochanteric fractures, and each has its own advantages. Among them, PFNA has a wide range of applications and relatively simple surgical operations, while PCCP is suitable for patients with poor surgical tolerance. Therefore, a comprehensive evaluation should be carried out according to the patient's age, fracture type, physical condition, and other factors, so as to select an appropriate surgical plan for internal fixation. The shortcomings of this study are that the sample size of the research object is small and it is a single-center study. Further studies with large samples and multiple centers are needed.

## Figures and Tables

**Figure 1:** Preoperative and postoperative X-ray images of left femoral intertrochanteric fracture with PCCP. (a) Preoperative left hip joint frontal radiograph. (b) Preoperative 3D CT reconstruction. (c) PCCP postoperative left hip joint frontal radiograph. (d) PCCP postoperative left hip joint lateral radiograph.

**Table 1:** Comparison of general data between the two groups.

Group	N	Age	Gender		Causes of injury			Fracture type		
			Male	Female	Car accident	High-altitude falling	Crash	A1	A2	A3
PFNA group	51	69.12 ± 9.13	27	24	9	8	34	16	16	19
PCCP group	47	67.06 ± 10.28	24	23	8	8	31	15	18	14
*t/χ * ^*2*^		1.050	0.035		0.034			0.745		
*P*		0.296	0.853		0.983			0.689		

**Table 2:** Comparison of intraoperative indicators between the two groups ($\bar{x}\pm s$, *n* = 98).

Group	N	Operation time (t/min)	Intraoperative blood loss (V/ml)	Postoperative drainage volume (V/ml)
PFNA group	51	63.36 ± 21.52	153.25 ± 32.68	68.19 ± 26.28
PCCP group	47	69.15 ± 18.38	58.69 ± 48.64	25.23 ± 16.10
*t*		−1.43	11.38	9.66
*P*		0.16	<0.01	<0.01

**Table 3:** Comparison of postoperative indicators between the two groups ($\bar{x}\pm s$, *n* = 98).

Group	N	Fracture healing time (t/week)	Time of weight-bearing (t/week)	Postoperative Harris score of hip joint function
PFNA group	51	17.2 ± 1.8	3.83 ± 1.20	84.68 ± 3.16
PCCP group	47	16.3 ± 2.9	4.35 ± 1.10	83.49 ± 4.05
*t*		1.86	−2.23	1.63
*P*		0.066	0.028	0.11

**Table 4:** Comparison of postoperative complications between the two groups (*n*, %).

Group	N	Delayed healing	Femoral neck nail cutting	Coxa vara	Nonunion of fracture	Total complications
PFNA group	51	1	2	1	0	4 (7.84)
PCCP group	47	1	3	0	1	5 (10.64)
*χ * ^*2*^						0.274
*P*						0.659

## Data Availability

The data can be obtained from the corresponding author upon reasonable request.
